The article "Induction of Interferon-Stimulated Genes by IRF3 Promotes Replication of Toxoplasma gondii" was retracted in 2024. Reasons: errors in the images; duplicated images; overlap with earlier publications; original data or images not available.

# Induction of Interferon-Stimulated Genes by IRF3 Promotes Replication of *Toxoplasma gondii*

**DOI:** 10.1371/journal.ppat.1004779

**Published:** 2015-03-26

**Authors:** Tanmay Majumdar, Saurabh Chattopadhyay, Evgeny Ozhegov, Jayeeta Dhar, Ramansu Goswami, Ganes C. Sen, Sailen Barik

**Affiliations:** 1 Center for Gene Regulation in Health and Disease, and Department of Biological, Geological and Environmental Sciences, College of Sciences and Health Professions, Cleveland State University, Cleveland, Ohio, United States of America; 2 Department of Molecular Genetics, Lerner Research Institute of the Cleveland Clinic, Cleveland, Ohio, United States of America; Cornell University, UNITED STATES

## Abstract

Innate immunity is the first line of defense against microbial insult. The transcription factor, IRF3, is needed by mammalian cells to mount innate immune responses against many microbes, especially viruses. IRF3 remains inactive in the cytoplasm of uninfected cells; upon virus infection, it gets phosphorylated and then translocates to the nucleus, where it binds to the promoters of antiviral genes and induces their expression. Such genes include type I interferons (IFNs) as well as Interferon Stimulated Genes (ISGs). IRF3-/- cells support enhanced replication of many viruses and therefore, the corresponding mice are highly susceptible to viral pathogenesis. Here, we provide evidence for an unexpected pro-microbial role of IRF3: the replication of the protozoan parasite, *Toxoplasma gondii*, was significantly impaired in IRF3-/- cells. In exploring whether the transcriptional activity of IRF3 was important for its pro-parasitic function, we found that ISGs induced by parasite-activated IRF3 were indeed essential, whereas type I interferons were not important. To delineate the signaling pathway that activates IRF3 in response to parasite infection, we used genetically modified human and mouse cells. The pro-parasitic signaling pathway, which we termed PISA (Parasite-IRF3 Signaling Activation), activated IRF3 without any involvement of the Toll-like receptor or RIG-I-like receptor pathways, thereby ruling out a role of parasite-derived RNA species in activating PISA. Instead, PISA needed the presence of cGAS, STING, TBK1 and IRF3, indicating the necessity of DNA-triggered signaling. To evaluate the physiological significance of our in vitro findings, IRF3-/- mice were challenged with parasite infection and their morbidity and mortality were measured. Unlike WT mice, the IRF3-/- mice did not support replication of the parasite and were resistant to pathogenesis caused by it. Our results revealed a new paradigm in which the antiviral host factor, IRF3, plays a cell-intrinsic pro-parasitic role.

## Author Summary

Interferon Regulatory Factor 3 (IRF3) is an essential transcription factor for the expression of antiviral genes, including type I IFNs and ISGs. The coordinated action of the ISGs leads to the inhibition of one or multiple steps of viral life cycle. In contrast to the well-known antiviral function of IRF3, we report here an unexpected pro-parasitic role of IRF3 in supporting the replication of the protozoan parasite, *Toxoplasma gondii*, in both cells and mice. The IRF3-deficient mice did not support *T*. *gondii* replication and, therefore, were protected from *T*. *gondii*-induced pathogenesis. The novel pro-*Toxoplasma* role of IRF3 was type I IFN-independent, but required its transcriptional function that induced the effector ISGs. Using cells deficient in known components of the IRF3 activation pathways, we have delineated the nature of the pro-parasitic signaling pathway, which we named ‘PISA’. Our detailed genetic and biochemical analyses revealed that PISA is activated by a *T*. *gondii*-triggered cytoplasmic cGAS/STING/TBK1-dependent pathway that activates IRF3 for the induction of the pro-parasitic ISGs.

## Introduction

*Toxoplasma gondii*, an obligate intracellular protozoan, is responsible for severe Toxoplasmosis [1]. Roughly one-third of the world's population is infected with *T*. *gondii*, which may lead to a mononucleosis-like syndrome with fever, lymph node enlargement, asthenia and headache. *T*. *gondii* is a major cause of blindness [1], and infection in pregnant women, transmitted transplacentally, can cause congenital fetal toxoplasmosis, leading to miscarriage, microcephaly, hydrocephalus, and seizures. To date, there is no vaccine against *T*. *gondii* for human use and no permanent cure for chronic toxoplasmosis; moreover, therapies such as pyrimethamine and clindamycin have significant side effects, including bone marrow suppression, rashes, and male infertility [2,3]. *T*. *gondii* evades adaptive immunity by transforming into dormant cysts that cause an asymptomatic chronic infection [4]. For this reason, the innate immune response of the host against *T*. *gondii* has received considerable attention, focused almost exclusively on cells of the immune system, such as macrophages and dendritic cells (DCs), and several key cytokines produced by these cells in response to *T*. *gondii* infection [5–10]. In contrast, little is known about the innate immune response that *T*. *gondii* elicits in non-immune cells, such as the epithelia, fibroblasts, the central nervous system (CNS) and ocular cells, which together represent important host organs for the parasite. In the current study, we investigated the role of the type I interferon (IFN) system, the most prominent antiviral innate immune response, in *T*. *gondii* infection of cells of immune and non-immune origins.

Microbial infection of mammalian hosts elicits a variety of immune responses that are temporally regulated. An early response is the activation of the innate immune signaling pathways that lead to the transcriptional induction of many cellular genes, including those encoding cytokines; the cytokines are then secreted and act upon as yet uninfected cells to forearm them against oncoming microbial infection. The IFN system is a good example of such a circuitry [11], whereby virus infection induces the synthesis of type I IFN that is secreted and activates immune cells to eliminate the infected cells. In addition, IFN can directly induce an antiviral state in a cell by inducing hundreds of genes, called IFN-stimulated genes (ISG), which encode intracellular proteins, some with the ability to interfere with different stages of virus replication. Surprisingly, ISGs can also be induced by many other signaling pathways activated by microbial infection, without any involvement of IFN, indicating a much broader physiological role of these genes [12].

Much is known about how ISGs are induced by microbes. Microbial pathogen-associated molecular patterns (PAMP) are recognized by cellular pattern recognition receptors (PRR), such as membrane-bound Toll-like receptors (TLR), cytoplasmic RIG-I-like receptors (RLRs), and various cytoplasmic DNA receptors [13,14]. One such receptor, STING, can be activated either by direct DNA-binding or by cyclic dinucleotides produced by the cyclic GMP-AMP synthase (cGAS), which is also activated by cytoplasmic DNA [15–19]. The PRRs use adaptor proteins, such as MyD88, TRIF or MAVS, to assemble different multi-protein signaling complexes, including specific protein kinases. One such protein kinase is TBK1, used by TLR3, TLR4, RLRs and STING to directly phosphorylate the latent transcription factor, IRF3, and activate it [20]. Activation causes nuclear translocation of IRF3, where it induces transcription of ISGs by binding to a specific promoter sequence, called ISRE. Thus, any signaling pathway that can activate TBK1 and IRF3 has the ability to induce ISGs. Other genes, such as that of IFN-β itself, need in addition to IRF3, other transcription factors for induction. Because the ISRE is recognized by all nine members of the IRF family, some signaling pathways use other IRFs to induce ISGs. For example, type I IFN-signaling uses a transcription complex containing IRF9 for this purpose. Thus, in an infected cell, ISGs are directly induced by IRF3, but concomitant synthesis of type I IFN can reinforce the ISG induction.

Here, we report that ISG induction by IRF3 is not only not detrimental to the parasite but it actually promotes efficient *T*. *gondii* replication, in cell cultures or in mice, although type I IFN itself has no role in it. We present evidence that this novel interaction between the parasite and IRF3, which we have termed "parasite-IRF3 signaling activation" (PISA), is achieved by parasite-mediated activation of TBK1 through the cGAS/STING pathway.

## Results

### Efficient replication of *T*. *gondii* requires host IRF3

To investigate whether the type I IFN system regulates the replication of unicellular parasites, we used the virulent *T*. *gondii* RH strain as a model, and measured parasite replication by immunoblot of parasitic SAG1 protein as well as quantitative PCR (qPCR) of the parasitic genomic DNA. Two types of mouse cells, mouse embryonic fibroblasts (MEFs) and bone marrow-derived DCs (BMDCs), and two human cell lines, HT1080 (fibrosarcoma) and M17 (neuroblastoma), were used, and in all cell types *Tg*SAG1 expression increased over time after parasite infection. Using this assay, we observed that *T*. *gondii* RH replicated poorly in cells deficient in IRF3 (Fig. 1A, 1B, 1C; S1 Fig.). Specifically, in MEFs (Fig. 1A) and BMDCs (Fig. 1B) from IRF3 -/- mice, or in human cells in which IRF3 was knocked down by shRNA (KD) (Fig. 1C), *T*. *gondii* replicated poorly. Expression of recombinant IRF3 in the HT1080 KD cells improved their ability to support parasite replication (Fig. 1C).

**Fig 1:** *T*. *gondii* replication is stimulated by IRF3. **A/B/C,** Three types of cells (MEF: mouse embryonic fibroblasts, DC: mouse dendritic cells, HT1080: human fibroblasts) were infected with *T*. *gondii* RH (a virulent type I strain). Total infected cell proteins at the indicated times post-infection were analyzed by immunoblotting to detect *T*. *gondii* SAG1 protein. U = uninfected cell control. The IRF3-deficient (KO = knockout; KD = knockdown with stably expressed shRNA) cells were compared with the corresponding wild type (WT), or with IRF3- restored, cells as noted. Parasite growth was also quantified by qPCR of genomic DNA using the invariant ITS-1 primers and normalized against GAPDH. **D,** Use of Tet (Dox)-off IRF3 expression system (Clone 10 cells) shows parasitic growth kinetics in response to IRF3. Immunoblot of the V5-tagged Tet-regulated recombinant IRF3 (top panels), *T*. *gondii* SAG1 (middle panels), and control actin (bottom panels) are shown. Left: Poor parasite growth in IRF3-repressed cells. Right: Growth kinetics of the parasite in the Clone 10 cells, in which IRF3 was induced by the withdrawal of Dox. In all panels, actin serves as the loading control. V5-IRF3 was detected by anti-V5 antibody.

To gain an understanding of the kinetics of IRF3 action, we used an engineered cell line, Clone 10, expressing recombinant V5-tagged IRF3 under Doxycycline (Dox) control [21]. To perform this experiment, we first determined the inhibitory concentration of Dox against *T*. *gondii*. Both the Western blot and the quantification of parasitic DNA showed an IC_50_ of 10–12 μg/ml in HT1080 host cells under our growth conditions (S2 Fig.), and essentially no inhibition at 1 μg/ml, the concentration of Dox we used to shut-down IRF3 expression in Clone 10 cells. When grown in the presence of Dox (1 μg/ml), these cells did not express IRF3 and did not support efficient *T*. *gondii* replication (Fig. 1D, left). Removal of Dox resulted in the appearance of IRF3 protein around 18 h and promoted robust *T*. *gondii* growth that closely followed on the heels of IRF3 appearance (Fig. 1D, right), consistent with parasitic growth stimulation by IRF3.

We further confirmed the stimulatory role IRF3 on *T*. *gondii* by two independent techniques: microscopy and flow cytometry, both of which clearly revealed stunted parasite replication in the IRF3-/- cells. In confocal microscopy, more parasites are seen the PVs in the wild type MEFs than in the IRF3-/- MEF at any time point of infection (Fig. 2A). For flow cytometry (Fig. 2B), we set the baseline to detect cells containing two or more parasites. With this gating, nearly all initially infected WT BMDCs scored as positive (30.91% of total, matching the m.o.i. of 0.3), whereas the number was significantly lower (6.28%) in the IRF3-/- BMDCs (Fig. 2B). When gated for 1 parasite per cell, KO and WT cells showed the same percentage of parasite-positive cells (30–33% of the total population), which was equal to the m.o.i (as shown for WT) (Fig. 2B). These results also indicated that IRF3 deficiency affected the intracellular replication of the parasite, but not the entry or the formation of PV.

**Fig 2:** IRF3 facilitates intracellular *T*. *gondii* replication regardless of parasite virulence type. **A,** Stunted parasite replication in IRF3 -/- cells. Isogenic wild type and IRF3 -/- MEF cells were infected by *T*. *gondii* RH at an m.o.i. of 0.2, and at the indicated times (4, 18, 24 h) stained for parasites (green), cytoplasmic actin (red) and nucleus (DAPI, blue) and visualized by confocal microscopy. For each sample, several individual PVs are shown; number of parasites in 12–14 PVs was counted and the mean ± SD values are shown. **B,** Flow cytometry measurement of parasite growth. DCs isolated from wild type and IRF3 -/- mice were infected with *T*. *gondii* RH at 0.3 m.o.i., and cells were permeabilized and dual-stained for CD11c and parasitic SAG1 at 18 h post-infection, with uninfected wild type cells as control. Gating was set to count infected cells with 2 or more parasites per PV, as marked by contour plot (left), and the percentage of such cells in the total population is shown. **C,** IRF3 is important for optimal growth of diverse *T*. *gondii* strains. The indicated *T*. *gondii* strains, represented the three major types: GT1 (type I), ME49 (type II), and VEG (type III). Infection was performed as in Fig. 1A, and total DNA was isolated at the indicated times. The amount of *T*. *gondii* DNA was quantified by qPCR of the genomic DNA as in Fig. 1.

The experiments described thus far used *T*. *gondii* RH, a highly laboratory-passaged non-cyst-forming strain. To inquire if the need for IRF3 extends to other types of *T*. *gondii*, we tested the growth of three more strains by qRT-PCR, which showed that IRF3 is needed not only for RH, but also for another type I strain (GT1) as well as type II (ME49) and type III (VEG) strains, although the extent of IRF3-dependence varied (Fig. 2C).

Together, using four independent parasite growth analyses, e.g. immunoblot, qRT-PCR, flow cytometry and confocal microscopy, we demonstrated a specific role of IRF3 in augmenting *T*. *gondii* replication that is independent of host cell and parasite types.

### Cellular gene induction by IRF3 is essential for parasite growth

Although IRF3 is well known as a transcription factor, we have shown that it can trigger apoptosis by a transcription-independent mechanism [22]. To inquire which function of IRF3 is critical for supporting parasite growth, we capitalized on the fact that the transcriptional function but not the pro-apoptotic function of IRF3 absolutely requires the presence of HDAC6, which deacetylates β-catenin, an obligatory co-activator of IRF3-driven transcription [23]. *T*. *gondii* in fact replicated very poorly in HDAC6-/- MEF cells (Fig. 3A), reinforcing our conclusion that in order to support parasite replication IRF3 was acting as a transcription factor of its target genes. Indeed, in infected cells, there was strong induction of ISGs, as manifested by the presence of the ISG56 protein (Fig. 3B, upper half). ISG56 induction did not require induced IFN as an intermediate because in IFNAR-/- cells, which cannot respond to type I IFN, infection caused similar induction of ISG56; moreover, *T*. *gondii* replicated well in these cells (Fig. 3B, lower half). As stated above, IFN can also induce ISGs, but not its own gene. Hence, we treated IRF3 KO MEF cells, which supported *T*. *gondii* growth poorly, with exogenous IFN-β to induce the ISGs and then challenged them with the parasite. As shown, *T*. *gondii* could replicate efficiently in IFN-β-treated cells, even when the cells did not express any IRF3 (Fig. 3C). These results strongly suggest that one or more ISG-encoded proteins, induced by activated IRF3, facilitate parasite replication; however, type I IFN is not required for this action of IRF3, although it can substitute for IRF3 by virtue of the fact that IFN and IRF3 can induce the expression of an overlapping set of genes, the ISGs.

**Fig 3:** Requirement of IRF3-induced host genes for *T*. *gondii* replication. **A,** Infection and immunoblotting was performed with HDAC6 KO and wild type MEF cells. **B**, MEF cells (wild type or IFNAR KO) were infected with *T*. *gondii* and the indicated proteins were measured by immunoblotting. **C**, *T*. *gondii* growth measured in IRF3 KO MEF cells; where indicated, recombinant murine IFN-β (2,000 U/ml, R&D Systems) was added, and parasite was added 6 h later. Immunoblotting was performed as above. Where shown, parasite growth was also quantified by qPCR of genomic DNA, and ISG56 (Ifit1) mRNA was quantified by qRT-PCR as described before [66].

### PISA activates IRF3 by its TBK1-mediated phosphorylation

Activation of IRF3, as a transcription factor, requires phosphorylation of at least two of its serine residues (Ser396, Ser398 in human IRF3 and Ser388, Ser390 in mouse IRF3) [24]. The known signaling pathways activate IRF3 through its phosphorylation by the protein kinase, TBK1, which in turn is activated by signal-dependent auto-phosphorylation [25]. The same scenario held true for IRF3 activation in *T*. *gondii*-infected cells. IRF3 was phosphorylated upon infection in all cell lines tested and the phosphorylation was sustained, indicating the continuous presence of active IRF3 in infected cells (Fig. 4A, left). In all cases, endogenous TBK1 was also phosphorylated with similar kinetics (Fig. 4A, right). The need for the two target Ser residues, 396 and 398, was confirmed by using an IRF3 mutant in which they were mutated; in IRF3 KD cells, expression of wild type IRF3 promoted efficient replication of *T*. *gondii* but the mutant IRF3 was ineffective (Fig. 4B). Finally, the essential role of TBK1 was confirmed by using TBK1 KO cells, in which IRF3 was not phosphorylated and the parasite replicated poorly; however, expression of recombinant TBK1 in these cells caused IRF3 phosphorylation as well as efficient parasite replication (Fig. 4C).

**Fig 4:** IRF3 phosphorylation is essential for PISA and *T*. *gondii* replication. Parasite infection and growth analyses were performed as described in Fig. 1A. Immunoblotting detected the indicated proteins, including phospho-IRF3 (P-IRF3), using a phospho-Ser396-specific antibody. **A,** The cell lines used are indicated. **B,** IRF3 KD (knocked-down) HT1080 cell line or these cells, reconstituted with WT or 396/98AA mutant of IRF3, were used for *T*. *gondii* infection. **C,** The indicated TBK1 KO and FLAG-TBK1-restored MEFs were used for *T*. *gondii* infection. Where shown, parasite growth was quantified by qPCR of genomic DNA.

### PISA is TLR-independent

To identify the specific signaling pathway used by PISA, we used various knockout cell lines devoid of strategic signaling molecules (Fig. 5). Without the knowledge of the nature of the PAMP used by *T*. *gondii* to activate PISA, we tested the requirements of the major PRRs and their adaptor proteins (Fig. 5A). RLRs were ruled out, because PISA was activated in RIG-I KO cells, as manifested by *Tg*SAG1 synthesis and IRF3 phosphorylation (Fig. 5A, panel 2); the same was true for all TLRs that use MyD88 as the obligatory adaptor protein, since loss of MyD88 also had no effect on PISA (Fig. 5A, panel 3). TLR3 and TLR4 can signal via TRIF instead of MyD88; however, neither of these TLRs were required for PISA (Fig. 5A, panels 4, 5), thus indicating a potentially novel signaling branch in PISA-related cellular signaling.

**Fig 5:** Essential role of a TLR3/4-independent cGAS-STING signaling axis in PISA and optimal *T*. *gondii* replication. Parasite infection and growth analyses were performed as in Fig. 1A. **A,** MEFs (WT, RIG-I-/-, TLR3-/-) and primary macrophages (MyD88-/-, TLR4-/-) were used for comparing PISA (*Tg*SAG1 expression or IRF3 phosphorylation) upon *T*. *gondii* infection. **B/C,** STING-/- MEF cells (B) or human 293T cells (C) were transiently transfected with wild type or mutant (mt) FLAG-cGAS and/or HA-STING plasmids, and infected as shown. **D,** Parasite growth in various conditions used in the other panels, quantified by qPCR; error bars are from three data sets.

### STING / cGAS signaling pathway is essential for PISA

Since neither RLRs nor TLRs were needed for PISA, we tested the DNA-sensing STING pathway, and found that PISA is indeed defective in STING KO MEF cells and that parasite growth as well as phosphorylation of TBK1 and IRF3 in these cells could be enhanced by recombinant expression of STING (Fig. 5B). STING can directly respond to cytoplasmic DNA; alternatively, the enzyme cGAS is activated by this PAMP and produces cyclic dinucleotides (CDNs), which in turn activate STING. To distinguish between these possibilities, we resorted to 293T cells, which are known to express very little cGAS and STING [18]. As expected, these cells did not support *T*. *gondii* replication (Fig. 5C). Ectopic expression of either cGAS or STING alone could not promote parasite growth; however, co-expression of both proteins fully triggered PISA, supporting efficient *T*. *gondii* replication as well as TBK1 and IRF3 phosphorylation. In contrast to wild type cGAS, an enzymatically inactive mutant of cGAS failed to trigger PISA. These results suggest that cGAS recognizes a PAMP, possibly parasitic DNA, and produces a CDN that activates STING and consequently TBK1 and IRF3.

Since the naturally low level of STING in 293T cells appeared to correlate with poor *T*. *gondii* growth, we inquired whether this may be true for some other commonly used cell lines. We first quantified the STING mRNA levels in the following cell lines, which were either immortalized or cancerous: A549, H196, H1048 (all lung carcinoma cells), HeLa (cervical cancer), and three kinds of 293 cells (also known as HEK293, human embryonic kidney cells), viz. 293T (expressing the T-antigen) and two 293 cell lines of unknown origin, obtained from different laboratories (ours and Dr. George Stark's). Quantitative RT-PCR results (Fig. 6A) revealed that the STING levels in these cells varied widely; A549 and H196 contained the highest amount, the two 293 cell lines contained slightly lower levels, and H1048, HeLa, HME, and 293T contained very small amounts. While the mechanism of the natural variation in STING expression is unknown, these results reveal the diversity that may exist within established cell lines, even those bearing the same name. When tested for PISA in terms of *T*. *gondii* growth (Fig. 6B, 6C), there was a general correlation with STING expression. For example, A549 and H196 cells supported robust parasite growth, the two 293 cells supported moderate growth, and H1048, HME and 293T supported poor parasite growth. As seen by others [26–28], our HeLa cell line supported decent parasite growth (Fig. 6B), even though it had a low level of STING, lending further support to the variability of cell lines and the contribution of multiple host determinants besides STING in parasite replication.

**Fig 6:** STING levels and *T*. *gondii* replication in selected human cells. **A,** STING mRNA levels of the indicated cell lines, determined by qRT-PCR, were plotted. **B/C,** *T*. *gondii* RH growth in cell lines of diverse STING levels, measured respectively by Tg SAG1 immunoblot (panel B, with actin as loading control) and by qPCR of parasite DNA (panel C).

### IRF3 promotes parasite infection and resultant pathogenesis *in vivo*

Upon establishing the need of IRF3 for promoting parasite growth in cell culture, we wanted to determine whether the same is true *in vivo* as well. For this purpose, mice of different genetic backgrounds were infected with *T*. *gondii* by intraperitoneal injections, and their rates of survival were monitored. Infection by the parasite killed WT mice in a dose-dependent fashion; in contrast, IRF3-/- mice were quite resistant to death at every dose of infection tested (Fig. 7A). For example, at the lowest dose of 10 parasites per mouse, all WT mice either died or suffered severe weight loss by 15 days post infection, whereas none of the IRF3-/- mice died even after 25 days post infection. The pathogenicity in the WT mice correlated with weight loss (Fig. 7B), high parasite loads in the key organs tested, including spleen, liver and brain, whereas parasites were nearly undetectable in the same organs of IRF3-/- mice (Fig. 7C). Since IL-12 has been shown to be a protective cytokine in the mouse model of *Toxoplasma* infection, we tested its level in IRF3-/- and WT dendritic cells (DCs), following parasite infection in culture, as well as in the serum of the mice upon infection. Whereas WT DCs and wild type mice produced IL-12 in response to *T*. *gondii* infection, the levels were much higher when IRF3 was absent (Fig. 7D). When we tested IL-12 induction in nonimmune cell types, no post-infection induction of IL-12 could be detected in the non-immune cells, such as A549, MEF and M17 cells (S3 Fig.). Thus, IRF3 is needed for parasitic replication in a cell-intrinsic manner in many cell-types, although it is possible that the higher systemic IL-12 levels in the IRF3 KO animal, likely produced by infected immune cells, plays an important or even dominant role in the lower parasitic lethality. The higher level of IL-12 could be due to the non-transcriptional IL-12-suppressive role of IRF3, as shown in elegant recent studies [29, 30]. Recent studies have also revealed that three members of the IFN-γ-inducible p47 GTPase family are induced upon *T*. *gondii* infection in mouse; they are IGTP, IRG-47 and LRG-47 [29]. Of these, IGTP and LRG-47 play a role in resistance to acute *T*. *gondii* infection [29,30]. However, all three were expressed in similar amounts in *T*. *gondii*-infected WT and IRF3 -/- mice, as measured by qRT-PCR (S4 Fig.), suggesting that the parasite resistance of IRF3 -/- mice is unlikely due to overexpression of these IFN-γ-inducible GTPases.

**Fig 7:** *T*. *gondii* growth and virulence in mice is promoted by IRF3. **A,** C57BL/6 wild type (WT, red lines) and IRF3−/− (blue lines) mice (of the indicated number, *n*) were infected with 10 (O), 50 (□), or 100 tachyzoites (Δ) (the number of parasites are shown as well), and survival was monitored. **B,** Body weight profile of WT and IRF3-/- mice upon *T*. *gondii* infection. C57BL/6 wild type (WT, red lines) and IRF3 KO (blue lines) mice (10 mice in each group) were infected with *T*. *gondii* (number of parasites shown) and monitored for their body weight for the indicated time. Due to severe weight loss (>25% of the original), WT mice were withdrawn at various days of infection and were euthanized. **C,** Mice were infected with 10 parasites as in panel A, and the indicated organs from live animals were harvested on the days indicated, followed by DNA isolation and real-time qPCR. Relative quantification was performed using standard curve analysis of purified parasite DNA, and results were expressed as pg of parasite DNA per mg of total tissue DNA, as shown. **D,** Left panel: Bone-marrow derived DC from IRF3 -/- and isogenic WT mice were infected with *T*. *gondii* RH at m.o.i. 10 in tissue culture, and IL-12 released in the media were assayed by ELISA using a commercial kit (R&D Systems). Right panel: IRF3-/- and isogenic WT mice were infected 10 parasites as in panel A and IL-12 in the serum of the live animals was assayed by ELISA.

## Discussion

We have uncovered a new signaling pathway, PISA, which is activated in mammalian cells upon infection with *T*. *gondii and* follows the scheme: Parasitic PAMP → cGAS → STING → TBK1 → P-IRF3 → ISG(s) → Parasite replication (Fig. 8). All the cellular proteins of the PISA pathway have been previously identified as signaling components of the host’s innate immune defense responses that protect it from viral or bacterial infection. In contrast, PISA is pro-microbial, not anti-microbial, and hence, should not be viewed as the host’s defense response; rather, it is the first example of a parasite co-opting an innate antiviral pathway for its replication. It remains to be seen whether this new paradigm is true for other intracellular protozoa as well. It is interesting to note that type I IFN was not needed for efficient parasite growth indicating that intracellular proteins, induced by IRF3 in the infected cells, promote this process.

**Fig 8:** Our working model for PISA. In this model, a parasitic PAMP (possibly DNA) is sensed by the PRR, cGAS; the CDN product of cGAS then activates the STING-TBK1 kinase complex, which phosphorylates IRF3. The phospho-IRF3 translocates into the nucleus and leads to the induction of specific, parasite-friendly host gene(s), which facilitate *T*. *gondii* replication, thereby causing pathology and death.

A recent study [31] concluded that intracellular death of *T*. *gondii* results in the release of its nucleic acids, leading to the activation of RNA or DNA receptors, thereby activating IRF3 and inducing IFN-β. Pioneering studies by Beiting et al [32] recently showed that in macrophages, heat-killed *T*. *gondii* induce ISGs more efficiently than live parasites. The loss of this induction in TLR3 -/- macrophages suggested that a *T*. *gondii* RNA, perhaps released by phagocytosis of the dead parasites, is the PAMP. We do not know if a fraction of the parasites in our preparation was dead, but it appears that UV-killed and heat-killed parasites interact differently with the host. We cannot rule out a contribution of RNA in PISA, but the lack a role of TLR3 and the need for cGAS suggest that DNA is likely the major PAMP.

Although the exact structural features of the DNA recognized by the cytoplasmic DNA sensors remain to be defined, unmethylated DNA of prokaryotic pathogens is a major PAMP. Interestingly, genomes of three *Apicomplexa* parasites, namely *Plasmodium falciparum*, *T*. *gondii* and *Cryptosporidium parvum*, contain very low or little methylation [33,34]. Purified genomic DNA of *P*. *falciparum* and *P*. *berghei* in fact activates the STING pathway [35] and type I IFN in an IRF3-dependent manner [36]. A new concept of PAMP, named 'viability-associated PAMP' or vita-PAMP, has been defined as an entity generated by viable pathogens and not by dead ones. Although the vita-PAMP of cytoplasmic bacteria was identified as mRNA generated from bacterial transcription [37], any *de novo* synthesized PAMP could potentially be a vita-PAMP. This concept may also hold true for *T*. *gondii* since we have observed that UV-inactivated, non-replicative parasite is unable to activate PISA. Unfortunately, our knowledge of the molecular exchange between the parasite and its host is highly limited. Nonetheless, an increasing number of *T*. *gondii* macromolecules are found to access the host cytoplasm, such as kinases and pseudokinases, injected into the host cytoplasm promptly after parasitic invasion, whereby they regulate specific host signaling pathways [38–49]. The parasitic rhoptry kinase (ROP16) and the rhoptry protein phosphatase 2C (PP2C) actually travel all the way to the host nucleus and likely regulate host gene expression [40,45]. As mentioned, it will be important to know if infecting parasites actually release DNA or RNA at any stage of growth and whether they reach the host cytoplasm to activate the cGAS-STING pathway.

We provide evidence that PISA promotes parasite replication but do not know whether additional pathways are also stimulatory. It remains possible that genes induced by other transcription factors, such as NF-κB and AP-1, that are known to be activated by STING signaling [50], co-operate with IRF3-induced genes in promoting parasite replication. A distinct feature of PISA is that it requires the adaptor protein, STING, and it appears that STING and TBK1 form a signal-dependent complex that activates IRF3; indeed, STING has been reported to bind and activate TBK1 *in vitro* [51].

Recent studies have shown that under certain conditions *T*. *gondii* is highly vulnerable to autophagy [52] and, in the absence of a documented apoptotic cascade in *T*. *gondii*, autophagy has been suggested to be the primary mechanism of programmed cell death in *T*. *gondii* and potentially other related parasites. It is tempting to speculate that parasite-induced ISGs suppress an autophagic response that might otherwise be triggered by a host defense mechanism.

PISA appears to be stimulatory to *T*. *gondii* replication in all human and mouse cell lines and primary cells that we tested. More importantly, without IRF3 and PISA, the parasite replicated poorly and was poorly pathogenic in mice. Pathogenesis in *T*. *gondii*-infected mice has been shown to be indirectly inhibited by IRF3 through its action on specific cytokine synthesis. Thus, in this context, IRF3 inhibits pathogenesis by *T*. *gondii*, in contrast to the cell-intrinsic pro-parasitic effect of IRF3 reported here. Not surprisingly, in IRF3-/- mice, the latter effect was overriding and little pathogenesis was observed because the parasite could not replicate in infected cells of these mice. We established the pivotal role of IRF3 and PISA in inducing ISGs to promote parasite replication but they can also be induced by many other pathways, activated by other stimulants that do not use IRF3. For example, the IFN-activated Jak-STAT pathway uses IRF9 whereas TLR7 and TLR9 use IRF7 to induce the same genes. Thus, even in the absence of IRF3, if IFN synthesis is induced by any viral or bacterial infection, circulating IFN will induce ISGs systemically and facilitate efficient *T*. *gondii* replication. Even for WT mouse, IFN produced by prior viral infection will make it a better host for subsequent *T*. *gondii* infection because the as-yet uninfected cells will already be loaded with ISG products. Therefore, in the natural context, viral or bacterial infection of an organism may set it up to be a better host for *T*. *gondii*.

The ISGs have so far been studied in the context of their specific antiviral activities; this report reveals an unexpected new facet of their physiological significance in promoting microbial growth. The new knowledge can, in principle, be exploited to inhibit toxoplasmosis; inhibitors of any components of PISA, including IRF3 and ISGs, will be attractive candidates for this purpose. For good reasons, much of the related research so far has focused on formulating potent agonists of TLR and RLR signaling to boost the innate immune response and host defense [53]. However, inhibitors for these pathways are also known; for example, we discovered several inhibitors of ISG induction by TLR3 through the screening of a chemical library [54]. A similar approach can be taken to identify small molecule inhibitors of PISA, which can target multiple ISGs that may be involved in promoting various steps of parasitic cell division [55].

## Materials and Methods

### Cells and reagents

H196, H1048, HME, and HEK293 cell lines were kindly provided by Dr. George Stark, Lerner Research Institute (LRI). All cells, with the exception of the primary macrophages and DCs, were grown in Dulbecco's minimum essential media (DMEM) supplemented with 10% FBS (fetal bovine serum), 20 mM L-glutamine, 100 U/mL of penicillin and 100 μg/mL of streptomycin (Life Technologies). Primary bone-marrow-derived DCs were obtained as follows. Bone marrow from the femurs and hind legs of mice of the appropriate genotype was collected in 1 ml of RPMI1640 medium (without serum) and single cell suspensions were made using 26G needle and syringe. Cells were washed twice with RPMI by centrifugation at 5,000 x g for 10 min in at 4°C, resuspended in RPMI containing 10% FBS, recombinant GM-CSF (PeproTech; Cat# 315–03) (10 ng/ml) and recombinant IL-4 (eBioscience; Cat# 14-8041-62) (10 ng/ml), and then grown for 8 days. The mature DCs were resuspended in RPMI plus 10% FBS and transferred to appropriate multi-well plates for infection with *T*. *gondii*. The details of the Clone 10 cells were described before [21]. Briefly, these cells were generated from the parental HT1080/shIRF3 cells by expressing N-terminally V5-tagged human IRF3, subcloned into pTRE2hyg vector (Clontech) and co-transfected with pTet-Off (Clontech). The resultant cells were selected against G418 (400 μg/ml), puromycin (1 μg/ml), and hygromycin (100 μg/ml). Where mentioned, MEF cells were treated with murine IFN-β (R&D Systems). Primary antibodies were obtained against the following: FLAG, HA and V5 epitope tags (Millipore), SAG1 and actin (Santa Cruz Biotechnology sc-52255, sc-8432, respectively), P-IRF3 (Ser 396), IRF3, P-TBK1 (Ser 172), TBK1 (Cell Signaling mAb #4947, mAb #4302, mAb #5483, #3013, respectively), and murine ISG56 (LRI Hybridoma Core). cGAMP (3'3' cyclic GAMP) was from Invivogen. Lipofectamine 2000 and Lipofectamine LTX with Plus reagent were from Invitrogen/Life Technologies.

### Plasmids and transfection

N-terminally V5-tagged human IRF3 and the deletion mutants were described before [22]. N-terminally HA-tagged STING and N-terminally Flag-tagged TBK1 were used for transfection experiments. Flag-tagged wild type (WT) cGAS and its enzymatically defective mutant were kindly provided by Robert Silverman (LRI). Human cell lines were transfected using Lipofectamine 2000, and mouse cells (MEFs), with Lipofectamine LTX with Plus reagent. Unless otherwise stated, 0.8 μg plasmid was used for transfection per 5 x 10^5^ cells (each well of a 12-well plate) using the manufacturers' instructions. After 8 h post transfection, cells were infected with *T*. *gondii* at an MOI of 2.

### Gene knockdown experiments

IRF3 knockdown HT1080 cells were described previously [22,56]. Briefly, these cells were generated by lentivirally expressing the shRNAs against the 5’ and 3’ UTRs of human IRF3 and selecting the resultant transduced cells under G418. These cells were used to express IRF3 by transfecting a cDNA of human IRF3 without the UTR. Clone 10 cells were described before and were derived from these parental cells.

### Growth of *T*. *gondii* stock and infection of cells

All *T*. *gondii* strains were grown in hTERT-immortalized human foreskin cells as described before [57,58] and purified by differential centrifugation (3,000 x g, 10 min), followed by filtration through 3 μm Whatman filter. Parasites were resuspended in phosphate-buffered saline, counted in a hemocytometer under microscope, and used for infection of cells at an MOI of 2, as described in Fig. legends. The infected cells were processed for immunoblot as described later. All experiments in this paper, except those indicated in Fig. 2C, used the *T*. *gondii* RH strain, which is a highly virulent, type I strain.

### Quantitative RT-PCR analyses

RT-PCR primers for cGAS and STING (Fig. 6A) were kind gifts of Dr. George Stark. Real-time qRT-PCR was performed as described with the following primer pair, against the ITS-1 region conserved in all *T*. *gondii* strains [59]: AATATTGGAAGCCAGTGCAGG (forward), CAATCTTTCACTCTCTCTCAA (reverse). Results were normalized against GAPDH gene, amplified with the following primers: CTGGAAAACCCTGCCAAATA (forward), TGCTCAGTTTAGCCCAGGAT (reverse). The primers for IGTP and LRG-47 have been described [60,61]; those for IRG-47 (GenBank M63630.1), designed by us, were: GCCAAACCCATAGCTTTCAAG (forward) and GAAATCAAACGCACCCAGATC (reverse). PCRs were setup in a final volume of 20 μl using 5 ng of template DNA, 200 ng of each primer and 1x of the iQ SYBR Green Supermix (BioRad). Quantitative RT-PCR analysis was performed on a DNA Engine Opticon 2 Real-Time Cycler (MJ Research). Primers directed against the *T*. *gondii* ITS-1 gene did not generate a product when the template genomic DNA was derived from organs of uninfected mice.

### Cell lysis and immunoblotting (IB)

Immunoblotting procedures were performed as described preciously [62,63]. Briefly, at the indicated times post infection (p.i.), cells were washed twice with PBS. For IB, cells were lysed by the addition of 1.5 x Laemmli sample buffer containing protease inhibitor (Roche, Product # 04693116001) and phosphatase inhibitor cocktails (Cell Signaling Technology, Cat# 5870). Cells were fully lysed by pipetting followed by sonication. Samples were heated at 95°C and equal amounts of proteins were analyzed on denaturing SDS-polyacrylamide gels. The proteins were transferred to PVDF Immobilon-P membrane (Millipore, Cat# IPVH00010) and probed with specific primary antibody followed by secondary antibody conjugated to horseradish peroxidase. Bands were visualized by chemiluminescence-based detection system (LI-COR Biosciences).

### Confocal microscopy

Cells (2.0 × 10^5^ /well) were plated onto cover glasses in 6-well plates, grown overnight (to ∼5 x 10^5^ cells), then infected with *T*. *gondii* at an m.o.i. of 0.2. At indicated times p.i., cells were fixed in ice-cold methanol for 5 min and permeabilized with PBS containing 0.1% Triton X-100. Fixed cells were blocked in PBS containing 1% BSA for 1 hr and labeled with anti-SAG1 as primary antibody (1:50) for 3 h, and Alexa Fluor 488-conjugated secondary antibody (1:200). Cytosol was stained with anti-actin antibody and Alexa Fluor 647-conjugated secondary. Nuclei were stained with DAPI. Cells were visualized at a 60× magnification in a Nikon A1RSI confocal microscope.

### Flow cytometry

DCs were prepared from wild type and IRF3-/- mice as described earlier and infected with freshly egressed RFP-expressing *T*. *gondii* RH strain at an m.o.i. of 0.3. At 18 h post-infection, the DCs were extensively washed to remove any free parasites, and 5 × 10^5^ cells were collected in 300 μl cold PBS and stained with anti-CD11c-FITC antibody (BD Pharmingen) for 1 hr at 4°. DCs were then washed with PBS, pelleted at 300 x g for 6 min at 4° C, fixed with 1% formalin, and analyzed for RFP-positive cells by flow cytometry in a FacsCanto II cell analyzer (BD Biosciences) using FlowJo software (Ashland, OR).

### Infection of mice with *T*. *gondii*

For *in vivo* infection, we used the IRF3-/- mice, as described before [23]. The stated number of RH parasites (e.g., 10, 50, or 100 as indicated in Fig. 7) in phosphate-buffered saline was intraperitoneally injected in mice [64,65]. For survival analyses, mice were monitored for the indicated time post-infection. For various tissue analyses, animals were sacrificed on the indicated days; organs were homogenized and total DNA isolated by the DNeasy Blood and Tissue kit (Qiagen, Valencia, CA). All animal procedures were approved by the Institutional Animal Care and Use Committee.

### Statistical analysis

Changes between treatment groups were analyzed by one-way ANOVA and by Student's *t*-test with Bonferroni correction. Numerical data were derived from three experiments, and results expressed as mean ± SEM or SD as stated (presented as error bars in graphs). P < 0.05 was considered significant.

## Supporting Information

S1 Fig Stimulation of *T*. *gondii* growth in human neuroblastoma M17 cells by IRF3. The M17 cells and its IRF3 knocked-down derivative were infected with *T*. *gondii* RH and the levels of the indicated proteins were quantified by immunoblot at 12, 18 and 24 h exactly as in Fig. 1A. Note the reduced parasite growth in the IRF3 knocked-down cells.
(TIF)

S2 Fig Test of doxycycline-sensitivity of *T*. *gondii*. HT1080 cells. The HT1080 cells in monolayer were infected with *T*. *gondii* RH at ∼1 m.o.i. under standard culture conditions (see Materials and Methods), in the presence of the indicated concentrations of doxycycline, and 48 h later cells were harvested and analysed as follows. (**A**) Immunoblot. Total cell lysates were subjected to immunoblot for *Tg*SAG1 and actin. (**B**) Total DNA from parallel cultures was purified and subjected to qPCR for Tg ITS-1 gene, and the results were plotted. Note the doxycycline IC_50_ of 10–12 μg/ml for *T*. *gondii* RH under these culture conditions in both assays.
(TIF)

S3 Fig Lack of detectable IL12 induction upon *T*. *gondii* infection of non-immune cell. IL-12 mRNA expressed in the indicated cell lines after 12 h of *T*. *gondii* infection, and in control uninfected cells, was quantified by qRT-PCR, and expressed as the ratio of GAPDH mRNA.
(TIF)

S4 Fig Similar induction of p47 GTPase genes (IGTP, IRG-47, LRG-47) upon *T*. *gondii* infection of WT and IRF3 KO cells. WT and IRF3 KO mice were infected with *T*. *gondii* as described in Fig. 7C and total mRNA was purified from the liver at 10 days later. qRT-PCR was performed with the primers described in Materials and Methods. Values were normalized against GAPDH mRNA as internal control, and fold inductions over the uninfected levels were plotted. Each bar represents average number from three mice ± SD.
(TIF)
